The article "Tumor microenvironment in non-melanoma skin cancer resistance to photodynamic therapy" was published in 2022. Journal: Front Oncol.

# Tumor microenvironment in non-melanoma skin cancer resistance to photodynamic therapy

**DOI:** 10.3389/fonc.2022.970279

**Published:** 2022-10-21

**Authors:** Paulina A. Cerro, Marta Mascaraque, María Gallego-Rentero, Manuel Almenara-Blasco, Jimena Nicolás-Morala, Juan Luis Santiago, Salvador González, Tamara Gracia-Cazaña, Ángeles Juarranz, Yolanda Gilaberte

**Affiliations:** ^1^ Department of Dermatology, Miguel Servet University Hospital, Instituto Investigación Sanitaria (IIS), Zaragoza, Aragón, Spain; ^2^ Department of Biology, Universidad Autónoma de Madrid, Madrid, Spain; ^3^ Department of Experminetal Dermatology and Skin Biology, Instituto Ramón y Cajal de Investigaciones Sanitarias, IRYCIS, Madrid, Spain; ^4^ Servicio de Dermatología, Hospital General de Ciudad Real, Ciudad Real, Spain; ^5^ Department of Medicine and Medical Specialties, Universidad de Alcalá, Madrid, Spain

**Keywords:** tumor microenvironment, non-melanoma skin cancer, resistance, photodynamic therapy, cancer-asssociated fiboroblasts, immune cells, mast cell

## Abstract

Non-melanoma skin cancer has recently seen an increase in prevalence, and it is estimated that this grow will continue in the coming years. In this sense, the importance of therapy effectiveness has increased, especially photodynamic therapy. Photodynamic therapy has attracted much attention as a minimally invasive, selective and repeatable approach for skin cancer treatment and prevention. Although its high efficiency, this strategy has also faced problems related to tumor resistance, where the tumor microenvironment has gained a well-deserved role in recent years. Tumor microenvironment denotes a wide variety of elements, such as cancer-associated fibroblasts, immune cells, endothelial cells or the extracellular matrix, where their interaction and the secretion of a wide diversity of cytokines. Therefore, the need of *designing* new strategies targeting elements of the tumor microenvironment to overcome the observed resistance has become evident. To this end, in this review we focus on the role of cancer-associated fibroblasts and tumor-associated macrophages in the resistance to photodynamic therapy. We are also exploring new approaches consisting in the combination of new and old drugs targeting these cells with photodynamic therapy to enhance treatment outcomes of non-melanoma skin cancer.

## Introduction

According to the Global Cancer Observatory, non-melanoma skin cancer (NMSC) has an annual incidence of 5.8% of the world population. In addition, in the last few years it has been observed an increase in its prevalence (between 3% and 7%) and it is estimated that it will continue in the coming years. The most common types include basal cell carcinoma (BCC) and squamous cell carcinoma (SCC) (1–3). The standard treatment options for NMSC include surgery, radiotherapy, chemotherapy as well as their combination (4, 5). However, within non-invasive treatments, photodynamic therapy (PDT) stands out, since it has become one of the therapeutic modalities that has grown the most in recent years, presenting numerous advantages over other treatments. PDT is a light-based therapeutic modality that involves administration of a tumor-localizing photosensitizing agent, which may require metabolic synthesis, followed by its activation with light of a specific wavelength. The mechanisms of action depend on the generation of singlet oxygen (^1^O_2_), through the excitation of the photosensitizer (PS), which transfers its excitation energy to the molecular oxygen in tumor tissues *via* triplet state. The necrotic, autophagy or apoptotic destruction of the tumor cells is induced by cytotoxic singlet oxygen and other secondary molecules such as reactive oxygen species (ROS) (4, 6) (**Figure 1**).

The article "Tumor microenvironment in non-melanoma skin cancer resistance to photodynamic therapy" was published in 2022. Journal: Front Oncol.

**Figure 1:** Mechanism of action on tumors in photodynamic therapy. The photosensitizer (PS) absorbs light and an electron moves to the first short-lived excited singlet state. This is followed by intersystem crossing, in which the excited electron changes its spin and produces a longer-lived triplet state. The PS triplet transfers energy to oxygen producing reactive singlet oxygen (^1^O_2_) and reactive oxygen species (ROS), which kill tumor cells. However, the tumor microenvironment protects the cancer cells against PDT through the interaction of its different constituents.

Moving on to other issues, despite the fact that the concept of tumor microenvironment (TME) has existed for more than a hundred years now, it has not been until recently that it has gained prominence (7). In this sense, tumors are not only constituted by cancer cells, but for a more complex intricate of diverse components (8). These TME constituents have been proved to be implicated in cancer cell survival, tumor development and therapeutic efficacy. Thereby, this tumoral stroma is composed by different cell types that fulfills their own role in these processes (9). Among them, fibroblasts, immune cells and endothelial cells are immersed in extracellular components, interacting with tumor cells. Moreover, a vascular network keeps nourished this amalgam of cells, where their crosstalk results in environment mediated drug resistance (10). These interactions proved to be involved in the effect of resistance of many tumors against different therapeutic strategies, specifically in PDT, are the object of the present review (**Figure 1**).

The article "Tumor microenvironment in non-melanoma skin cancer resistance to photodynamic therapy" was published in 2022. Journal: Front Oncol.

## Tumor microenvironment components

### Cancer-associated fibroblasts and cytokines

Fibroblasts are the main cell type present in the dermis. Because the dermis provides strength and flexibility to the skin, some of the principal functions of dermal fibroblasts are directly related to these abilities. Among others, wound healing and deposition of collagen and elastic fibers of the extracellular matrix (ECM) in connective tissue can be pointed out (11–13).

In the TME, normal fibroblasts suffer an activation process, acquiring specific characteristics and expressing differential markers such as vimentin, smooth muscle actin alpha (α-sma) and fibroblast activation protein (FAP) (14) (**Figure 2**). At this point, they receive the name of cancer-associated fibroblasts (CAFs) (15). Nevertheless, CAF populations have turned out to be heterogeneous, coexisting within the same tumor (such as inflammatory or myofibroblastic phenotypes) (16, 17). Because of this diversity, recent investigations have focused their efforts to study the broad amount of cytokines implicated in these changes (such as transforming growth factor beta (TGFβ), Interleukin-1 (IL-1) or integrins), as they are not only morphological, but also functional (18–21).

**Figure 2:** Role of CAFs, TAMs and TILs in the resistance to therapies. CAFs (cancer-associated fibroblast), TAMs (tumor-associated macrophages) and TILs (tumor infiltrated lymphocytes) produce cytokines that are taken up by tumor cells, producing changes in them. Epithelial mesenchymal transition (EMT), angiogenesis, quiescence and immune evasion, all factors that favor resistance to different treatments. CD8, cluster of differentiation 8; FAP, fibroblast activation protein; Foxp3, forkhead box P3; IL, interleukin; MCH-2, major histocompatibility complex 2; MMP, matrix metalloproteinases; PD-L1, programmed death-ligand 1; TGFβ, tumor growth factor; TNFα, tumor necrosis factor; VEGF, endothelial growth factor; α-SMA, smooth muscle actin alpha.

Related to these functional changes, the crosstalk between different CAF populations and tumoral cells has been long associated with resistance to therapies in different cancer types. In this sense, chemotherapy resistance (with compounds such as cisplatin, tamoxifen or gemcitabine) is the most studied one (22–25). One of the main mediators related to these resistance effects is TGFβ. This cytokine, in combination with many other molecules, plays a key role in CAF heterogeneity (26–30). In this sense, TGFβ modulates tumor progression and therapy response through CAF activation status, shape and invasiveness (31–33).

Within tumor progression, CAFs promote migration and invasion of tumor cells through a well-known process: the epithelial-mesenchymal transition (EMT) (34). In this regard, CAFs secrete a variety of activators that initiate the TGFβ cascade in epithelial tumor cells leading to a change in morphology and response, acquiring quasi-mesenchymal characteristics (35–40). On the other hand, not only CAFs modulate EMT but also tumor cells themselves through the expression of EMT factors that interact with the TGFβ signaling, such as FOXF2 or SOX9 (41–43) (**Figure 2**). Thus, the presence of these ones and similar markers constitutes an indubitable signal of malignant progression in several types of carcinomas (44, 45). Moreover, TGFβ secreted by CAFs also participates in the formation of vascular-like channels not only by endothelial cells, but also by tumor cells (46) (**Figure 2**).

The article "Tumor microenvironment in non-melanoma skin cancer resistance to photodynamic therapy" was published in 2022. Journal: Front Oncol.

On the other hand and as stated before, CAFs are able to modulate the response of tumoral cells to different therapies, generating resistance effects (47–53). Specifically, the main mechanism that prompts this phenomenon is the TGFβ-SMAD pathway, which can be modulated by different MAPKs (19, 54–58) More extensively, translocation of the SMAD complex to the nucleus targets specific genes such as p21 and p15, which are two potent inhibitors of the cyclin dependent kinases (CDKs), main regulators of the cell cycle (59–63). Thus, this provokes cell cycle arrest in the G1 phase as a consequence of the dysregulation of the G1/S checkpoint (57, 61, 64, 65). Consequently, this cell cycle arrest induces a dormant or quiescent state of tumoral cells which prevents their effective response to therapy, constituting an underlying mechanism of therapy resistance and tumor recurrence (66) (**Figure 2**). Moreover, p21 also stimulates the glutathione metabolism, which triggers an antioxidant response related to a drop in ROS levels (main effector in most conventional therapies) (53, 67). In this sense, the combination of therapies with compounds able to interrupt the TGFβ pathway could abrogate this cell cycle arrest, and hence, the resistance effect (66, 68).

### Tumor associated macrophages

Macrophages are one of the principal types of immune cells in innate immunity. They display different roles in pathogen phagocytosis antigen presentation and tissue regeneration. Despite its multiple beneficial functions, in a carcinogenic environment its recruitment could be detrimental. Tumoral context could induce a polarization in these cells, towards M1 antitumoral macrophages or towards M2 protumoral macrophages (69). These specific macrophages are defined as tumor associated macrophages (TAMs), which interact, modulate and influence tumor progression, invasion and metastasis. The main difference between them two is that antitumor agents act by releasing cytokines that promote adaptive immunity (IL-1, IL-6, TNF-α, NO, etc.) and have a high expression of MCH-2 (major histocompatibility complex 2) molecules, allowing the presentation of tumor antigens to cells of the immune system. In contrast, pro-oncogenic macrophages act by releasing anti-inflammatory cytokines (IL-4, IL-13, IL-10, TGFβ etc.), overexpressing PD-L1 (Programmed death-ligand 1), and expressing few MCH-2 molecules (70) (**Figure 2**).

The article "Tumor microenvironment in non-melanoma skin cancer resistance to photodynamic therapy" was published in 2022. Journal: Front Oncol.

Tumor associated macrophages influence tumor progression through secretion of cytokines such as IL-10, INF-γ and CCL5. These cytokines trigger the activation of JAK1/STAT1/NF-κB/Notch1, JAK/STAT3 β-catenin/STAT3 and PI3K/AKT signaling pathways, modulating tumor progression, stemness and metastasis (58, 71, 72) (**Figure 2**). However, TAMs do not always contribute to tumor progression. The balance between M1 and M2 polarization of them is critical to predict the prognosis of the patient (73–75).

Apart from being predictor of poor prognostic, TAMs are related to poor response to chemotherapy generating a resistance effect in colorectal cancer and glioblastoma models (76, 77) and to immune checkpoint inhibitors in prostate cancer (78). The modulation of this kind of cells may lead to a better response and tumor remission. However, it is hard to understand how they produce this effect. The blockade of molecules as PD-L1 and Stat6 with different antibodies leads to TAMs reprogramming, enhancing antitumor activity (79–81). mTOR inhibitors like Rapamycin and Metformin show the ability to modulate TAMs, boosting other therapies and controlling tumor progression (82, 83). Other compounds such as Chloroquine and its derivatives are, as well, modulators of TAMs polarization through an antitumoral phenotype, sensitizing tumor cells to chemotherapy (84, 85).

### Other immune cells present in the tumor microenvironment

Lymphocytes are the principal type of cell in adaptive immunity, they recognize specific antigens and produce a specific immune response. These cells are subdivided according to the expression of different markers such as CD3 (cluster of differentiation 3), CD25, CD4, CD8 or Foxp3 (forkhead box P3) exerting different responses against the pathogens (86). In a tumoral context, those tumor-interacting lymphocytes are defined as tumor infiltrated lymphocytes (TILs). TILs can modulate the development of the tumor depending on its features, which could be affected by the tumor at the same time. Specifically, high levels of cytotoxic CD8+ TILs infiltration tend to present antitumor activity and better outcomes for the patient (71, 87, 88). On the contrary, high levels of Foxp3+ regulatory T cells are strictly correlated with immunosuppression and pro-tumor activity triggering poor outcomes (89–91) (**Figure 2**).

The article "Tumor microenvironment in non-melanoma skin cancer resistance to photodynamic therapy" was published in 2022. Journal: Front Oncol.

B lymphocytes could also be part of the TME. It has been demonstrated that its presence is related with a higher CD8+ cells infiltration and, therefore, with a better prognosis (92, 93). However, this B cell appearance is not always beneficial, since these cells can also adopt a regulatory phenotype under the influence of myeloid-derived suppressor cells (MDSCs). Once with the regulatory phenotype, those cells produce cytokines with immunosuppressive effect, depleting CD8+ cells antitumor activity (94).

Myeloid-derived suppressor cells comprises a heterogeneous group of cells which have in common its derivation from immature myeloid cells and play an important role in cancer development, progression, invasion and setting of the pre-metastatic niche in different types of cancer (95). The protumoral activity derived from MDSCs is driven by several molecules present in the tumor as the macrophage migration inhibitory factor, B7 homolog 3 protein, also known as CD276, or signal transducer and activator of transcription 3 (STAT3) (96, 97). MDSCs could be modulated by different molecules and drugs in order to suppress their effects. Metformin, STAT 1 or the blockade of IL-6 and NLRP3 (NLR family pyrin domain containing 3) inflammasome can improve the clinical outcome and the prognosis of the patient (98–100).

Mast cell (MC) infiltration has been reported in a wide range of human and animal tumors particularly malignant melanoma and breast and colorectal cancer. The consequences of their presence in the TME remain unclear. Within the tumor, MC interactions occur with infiltrated immune cells, tumor cells, and ECM through direct cell-to-cell interactions or release of a broad range of mediators capable of remodeling the TME. MCs actively contribute to angiogenesis and induce neovascularization by releasing the classical proangiogenic factors including VEGF (vascular endothelial growth factor), FGF-2 (fibroblast growth factor), and IL-6, and nonclassical proangiogenic factors mainly proteases including tryptase and chymase (**Figure 2**). MCs may support tumor invasiveness by releasing a broad range of matrix metalloproteinases (MMPs) (101). 5-ALA-mediated PDT was associated with degranulation of MC and angiogenesis in oral premalignat lesions induced in rats (102).

Finally, the neutrophils also are associated with tumor progression. They are capable of establishing a pro-tumor microenvironment, being correlated to poor prognosis in some tumors such as lung cancer (103–105).

The article "Tumor microenvironment in non-melanoma skin cancer resistance to photodynamic therapy" was published in 2022. Journal: Front Oncol.

### Extracellular matrix

The extracellular matrix is a key factor in carcinogenesis, which offers structural and biochemical support for cellular components lowing it to influence cell communication, adhesion and proliferation (106). It consists of a network of macromolecules, including collagen, fibronectin, laminin and glycosaminoglycans (107, 108). Alteration in ECM components may be the basis for the tumor progression. For example, the laminin receptor expression plays an important role in SCC progression (109, 110); the loss of type IV collagen correlates with the poorly differentiated SCC (111) and fibronectin mediates cellular interactions with the ECM and it is important in cell migration (112). Matrix metalloproteinases (MMPs) are critical molecules for the EMT process because they degrade cell adhesion molecules and cell-ECM interactions, which are produced by both tumor and immune cells (106, 107). Finally, the ECM is also modulated by the action of CAFs through the secretion of soluble factors such as cytokines (113).

It should be noted that there is an interconnection between the different components of the EMT. TAMs are capable of producing differential responses in TILs depending on their polarization (114, 115). These TAMs could also be influenced by regulatory T cells, promoting a protumoral phenotype *via* repression of CD8+ secreted INF-γ (116). Also, CAFs have demonstrated marked effects on macrophages, attracting them and polarizing them to protumoral TAMs (117–119). In addition, CAFs, TAMs and TILs are providers of pro-angiogenic factors such as VEGF for the formation of a complex vascular network to meet the metabolic and nutritional needs of tumors (120–122).

## The tumor microenviroment as mediator of photodynamic resistance in non-melanoma skin cancer – Therapeutic opportunities

Photodynamic therapy not only targets neoplastic cells and tumor blood vessels, but also activates the immune system to induce inflammation and immune response to tumor cells (123). Although the intrinsic cellular mechanisms of resistance to PDT have been characterized, the emerging importance of the TME and the inflammatory/immune antitumor response is currently under investigation (123, 124). The specific role of CAFs and TAMs as an extrinsic mechanism of PDT resistance is attracting the attention for of researchers and is summarized in **Table 1**. Furthermore, although PDT has been extensively evaluated, both preclinically and clinically for the treatment of cancer cells, it has not been fully examined the concept of leveraging PDT to attack the tumor stroma in order to counteract therapeutic resistance induced by stromal signalling (149).

The article "Tumor microenvironment in non-melanoma skin cancer resistance to photodynamic therapy" was published in 2022. Journal: Front Oncol.

**Table 1:** Mechanisms of resistance to PDT caused by TME in NMSC and strategies to avoid it.

Effects of TME in PDT resistance	Strategies to improve PDT
Physical barrier for photosensitizers and intra-tumoral infiltration of immune cells	Disrupting the tumor extracellular matrix with hyaluronidase using dextran as a carrier (125)
Tumor hypoxia (126): Immunosuppressive effect by MDSC (123, 127)	Reduction of HIF-1α with curcumin (128) Delivering O2 to hypoxic tumors (129–131)
Responses of CAFs after PDT: Production of TGFβ-1 induces a quiescent in tumor cells after PDT (47, 132–134) Induction of tumor progression (135) Secretion of IL1β, which induces tumor promotion (136) Production of CXCL12, which avoids the contact between T cells and cancer cells (137)	Targeting CAFs: Reversion of CAFs phenotype by ALA (138) MAL + TGFβ inhibitor (47) Metformin + MAL inhibits TGFβ (139) ZnF16Pc-loaded ferritin nanoparticles eliminate CAFs (140, 141)
Suppression of tumor cell phagocytosis by M1 TAM (142, 143) M2 TAM exhibit pro-oncogenic properties (70): Releasing anti-inflammatory cytokines (IL4, IL13, IL10, TGFβ) Overexpressing PD-L1 Downregulation of MCH-2 molecules	Combination of PDT with drugs to promote M1 TAM polarization: Rapamycin (82) Metformin (83) Chloroquine (84, 85) Designing new PS for TAM, promoting M1 TAM over M2 TAM: Chloroaluminum sulfonated phthalocyanine (142, 144) Photofrin (143, 145, 146) Alginate-zinc (II) phthalocyanine conjugates (147) Mannose conjugated-chlorin (148)
Increase of degranulation of MC and angiogenesis (102)	Antihistamines (102)

ALA, aminolevulinic acid; CAFs, cancer-associated fibroblasts; CXCL12, C-X-C motif chemokine ligand 12; EMT, epithelial-mesenchymal transition; IL1β, Interleukin 1β; MAL, methyl aminolevulinate; MC, mast cell; MMP, metalloproteinases; NF-κB, Nuclear factor kappa-light-chain-enhancer of activated B cells; PDT, photodynamic therapy; PS, photosensitizer; TAM, tumor associated macrophages; TGFβ, tumor growth factor beta; TME, tumor microenvironment.

### CAFs and PDT

Studies on the role of fibroblasts in the effectiveness of PDT in neoplastic cells are infrequent, and most of them have been evaluated in pancreatic cancer. *Glidden et al.* observed greater resistance to PDT when pancreatic ductal adenocarcinoma cells were co-cultured with normal fibroblasts for 7 days in 3D models (150), while *Celli et al.* did not observe effects from normal fibroblasts in the effectiveness of PDT in pancreatic cancer cells (149). Also, *Chen et al.* did not appreciate significant differences using conditioned culture medium of CAFs in 2D and 3D cultures (151). The role of CAF-derived TGFβ-1 as an extrinsic factor has been identified in different cancers, including cutaneous squamous cell carcinoma (cSCC) and basal cell carcinoma (BCC), the two main types of NMSC, in which it can induce resistance to different therapies (47, 132–134). Recently, our group investigated the role of TGFβ-1 in the resistance process to PDT in NMSC cells, showed that the TGFβ-1 secreted by CAFs of SCC is capable of conferring resistance to PDT with methyl aminolevulinate (MAL) through the induction of a quiescence state, postulating TGFβ-1 as a target for PDT optimization (47) (**Figure 3A**).

The article "Tumor microenvironment in non-melanoma skin cancer resistance to photodynamic therapy" was published in 2022. Journal: Front Oncol.

**Figure 3:** Strategies for outcome PDT resistance generated by CAFs. **(A)** To inhibit TGFβ secretion; **(B)** To revert the CAFs phenotype by PDT; **(C)** To boost PDT at dermal level by UVA light; **(D)** To activate NLRP3 inflammasomes by PDT to induce an inflammation response by IL1β; **(E)** To direct PDT to CAFs using their components as targets, such as FAPs. FAP, fibroblast activation protein; IL1β, Interleukin 1β; NLRP3, NLR family pyrin domain containing 3; TGFβ, tumor growth factor beta.

Furthermore, although the selectivity of PDT for tumor cells has been widely reported, the effect of ALA-PDT on CAFs is not well understood. However, it has been shown that alterations in the TME, such as the emergence of CAFs, are necessary for tumor progression to invasive and metastatic SCC, stages resistant to PDT (135). *Li et al.* indicated the effect of PDT with 5-aminolevulinic (ALA) on SCC-CAFs, showing a revers of the activation of CAFs (a reduction in α-SMA, FAP expression and migratory capacity of these cell types) (138) (**Figure 3B**). An interesting field of study is the effect of CAFs on genodermatoses that predispose to skin cancer such as Gorlin-Golz syndrome (GS) and Xeroderma pigmentosum (XP). *Zamarron et al.* investigated the overexpression of α-SMA and vinculin in fibroblast from GS and XP patients, observing an increase in the expression of both markers as compared to healthy fibroblasts and thus considering that primary fibroblasts obtained from these patients could be potential CAFs (152). PDT is an interesting treatment option in these two genodermatoses that achieves high clearance rates and excellent cosmetic outcomes probably due to the susceptibility of GS and XP fibroblasts to PDT (153). The fact that these fibroblasts behave as CAFs is likely contributing to malignancy in this genodermatoses. On the other hand, since they are highly susceptible to MAL-PDT, it suggests that this approach could not only be relevant to treat the epithelial component of tumors or premalignant lesions but also the activated stromal cells. One mechanism that *Zamarron et al.* have proposed to improve the efficacy of PDT is a priming response elicited by UVA light (the one with the capacity to reach the dermis) that may enhance the effect of MAL-PDT (152) (**Figure 3C**).

The article "Tumor microenvironment in non-melanoma skin cancer resistance to photodynamic therapy" was published in 2022. Journal: Front Oncol.

On the other hand, there are several investigations showing that CAFs are mediators of inflammation in squamous cell carcinogenesis through the IL1β secretion. This cytokine has a dual role of tumor promotion and suppression. In this sense, *Nie et al.* preliminarily demonstrated that the NLRP3 inflammasome mediating IL1β production in CAFs contributes to the PDT effect with ALA on SCC (136) (**Figure 3D**). Thus, modulating the inflammatory response and knowing well the expression of cytokines produced by CAFs could be a mechanism to avoid tumor resistance to PDT.

Besides the different mechanisms previously described to combat extrinsic resistance to PDT induced by the tumor stroma, other possible strategies have been investigated. Among the different mechanisms proposed, highlights the use of nanomedicine. *Li et al.* found that a single chain viable fragment (scFv, sequence specific to FAP) and the PS ZnF16Pc-loaded ferritin nanoparticles (scFv-Z@FRT) can mediate efficient and selective PDT, leading to eradication of CAFs in tumors (140) (**Figure 3E**). This strategy has proven to be a new and safe CAF-targeted therapy and a novel way to modulate TME in order to enhance immunity against cancer. This is due to CAFs regulate C-X-C motif chemokine ligand 12 (CXCL12) secretion and ECM deposition, preventing physical contact between T cells and cancer cells (137, 141).. Finally, another strategy to combat resistance to PDT is the use of drugs that have a synergistic and adjuvant effect, such as the combination of PDT and the multi-kinase inhibitor cabozantinib for extensive desmoplasia in pancreatic ductal adenocarcinoma, which frequently associates with treatment resistance. Blocking EMT phosphorylation with adjuvant cabozantinib caused a significant improvement in PDT efficacy with benzoporphyrin derivative, most notably by elevating spheroid necrosis at low radiant exposures (154). Even drugs with other therapeutic purposes such as metformin with promising effects in SCC cells resistant to MAL PDT, could increase the response to this treatment (139). Since metformin inhibits TGFβ-1-mediated EMT in breast cancer (155) and in carcinoma cells of the cervix through the inhibition of mTOR/p70s6k signalling (156). In non-small cell lung cancer, a recent study has shown that metformin exerts antitumor effects such as inhibition of proliferation and invasion as well as control of EMT through inhibition of NF-κB (Nuclear factor kappa-light-chain-enhancer of activated B cells) (157). Finally, CAFs have been reported to play a role in inhibiting apoptosis, among other factors (158). However, to date, there are no data on the part of these proteins and PDT resistance.

The article "Tumor microenvironment in non-melanoma skin cancer resistance to photodynamic therapy" was published in 2022. Journal: Front Oncol.

### TAMs and PDT

Tumor associated macrophages also play complex but principal roles in the outcomes of PDT in malignant lesions Haga clic aquí para escribir texto.. The infiltration of M2 type TAMs to the neoplasm is associated with an increased risk of metastasis and tumor progression, due to the induction of angiogenesis and cell proliferation (159). The plasticity of TAMs can be used from a therapeutic point of view to generate more antitumor macrophages and destroy the neoplasm (70). TAMs have been shown to have a great capacity for the uptake of systemically administered PSs. *Chan et al.* used flow cytometry analysis and cell sorting to determine the content of a photosensitizer in the cellular fraction of a mouse colorectal carcinoma. Upon separating tumor-derived populations of high and low PS content, they identified macrophages among the cells with a high content (144). *Korbelik et al.* even showed that the amount of PS was greater in macrophages than in cells from the tumoral parenchyma (145). Macrophages M2 are selectively destroyed with PDT, and during the ensuing inflammatory reaction they are replaced with newly invading macrophages of M1 phenotype. Macrophages M1 have a principal role in the effect of PDT since they mediate in the removal of killed cancer cells and in the processing/presenting tumor antigens to T lymphocytes (160). The behavior of macrophages treated with PDT has been the subject of various studies. Macrophages treated with low doses of PDT seem to be activated and have greater activity, while those treated with higher doses lose their functionality (142). In addition, the macrophages treated with PDT generate a high amount of TNF-α, which entails the cytotoxic effect associated to this cytokine (146). Other mediators that are generated during PDT in the presence of TAMs and neoplastic cells are complement proteins (C3, C5 and C9), pentraxin, sphingolipids or toll-like receptors (TLR2, TLR4 and C3aR). All these molecules opsonize damaged tumor cells and facilitate phagocytosis by M1 TAMs (143).

The use of nanoparticles has become a strategy for the treatment of neoplasms. The development nanoparticles-based PDT against TAMs opens up new and more selective therapeutic pathways that can avoid resistance (161). TAMs express several receptors, including scavenger receptor A (SR-A), which can bind a variety of polyanionic ligands. Therefore, the conjugation of a PS with a polyanionic compound can act more selectively on them (162) (**Figure 4A**). Furthermore, alginate is a natural anionic polymer that has been combined with a PS known as phthalocyanine (1-[4-(2-aminoethyl) phenoxy]zinc(II) phthalocyanine) in a 0.1% gel presentation. The result is a low-cost photosensitizing molecule that is effective *in vivo* and *in vitro* against tumors of murine lines. Side effects were minimal and local, and the effectiveness over TAMs was high (147).

The article "Tumor microenvironment in non-melanoma skin cancer resistance to photodynamic therapy" was published in 2022. Journal: Front Oncol.

**Figure 4:** Strategies to eliminate TAM-2 by PDT. PS conjugation with TAMs receptors, such as **(A)** SR-A or **(B)** Manose receptors; **(C)** inhibition of HIF-1α, which promotes TAM-2. CD206, mannose receptor; HIF-1α, hypoxia factor 1; SR-A, scavenger receptor A; TAM-2, tumor associated macrophages 2.

Tumor associated macrophages overexpress CD206, a mannose receptor that is crucial for the role of macrophages in engulf, invasion and degradation of organism by endocytosis and phagocytosis (163). The use of mannose-conjugated chlorin (m-chlorin, photosensitizing substance) to target mannose receptors in TAMs has also been studied (**Figure 4B**). This PDT approach is a targeted therapy of TME TAMs to avoid their resistance, which induced a greater cell death in TAMs M2 (with mannose receptor) than TAMS M1 in cancer cells from the digestive tract (148). Finally, another strategy used to reduce TAMs-induced resistance is the use of curcumin as PS. Curcumin is a natural bioactive compound isolated from the rhizomes of Curcuma longa L., that exhibits great anti-tumor activity through the reduction of the levels of hypoxia factor 1 (HIF-1α) generated during PDT. HIF-1α promotes the M2 phenotype of macrophages and tumor survival, thus limiting the effectiveness of PDT (128) (**Figure 4C**). In the TME, uncontrolled cell proliferation avoid the ability to satisfy the oxygen demand from the preexisting blood vessels. Hypoxia has been found to directly regulate the expression of not only macrophages but also of other immune cells such as MDSCs (123, 127). In PDT, molecular oxygen is necessary, as a microenvironment of hypoxia could lead to treatment failure and drug resistance (126). Therefore, multiple nanomedicine-based strategies are being developed to circumvent hypoxia, such as hemoglobin oxygen carriers and cellular respiration inhibitions (129–131).

## Conclusion

Cancer not only has a malignant epithelial component but also a stromal with various components, such as fibroblasts, endothelial and inflammatory cells, which form an appropriate TME to promote tumorigenesis, progression, and metastasis. TME components have been found to influence the processes of resistance to various treatments, and photodynamic therapy is not spared. Several studies have linked resistance to this treatment to the presence of cancer and/or macrophages-associated fibroblasts, the two major components of the tumor microenvironment. To date, the importance of TGFβ-1 in the resistance process to PDT in NMSC cells has been demonstrated, as CAFs induce tumor progression and tumor promotion by IL1β after PDT, avoiding physical contact between T cells and cancer cells by CXCL12 after PDT, or showing how high dose of PDT suppress macrophages activity.

The article "Tumor microenvironment in non-melanoma skin cancer resistance to photodynamic therapy" was published in 2022. Journal: Front Oncol.

Although different mechanisms to prevent resistance to PDT have already been studied (**Table 1**), more strategies are needed to target this component to inhibit the tumor growth and prevent resistance to PDT in NMSC. In this sense, strategies based on nanomedicine to enhance PDT, as well as new photosensitizers or nano-sized photosensitizer, and the use of combined treatments could contribute to the development of future perspectives. Furthermore, the mechanism by which photodynamic therapy may produce an inflammatory response that favors tumor remission and thus future recurrences should be extensively studied.

## Author contributions

SG, YG, and AJ conceived the idea. PC, MM, MG-R, MA-B, JN-M, JS, and TG-C contributed to the preparation of manuscript and critically modified. MM and TG-C contributed in the preparation of figures. All authors contributed to the article and approved the submitted version.

## Funding

The work was supported by Spanish grants from Instituto de Salud Carlos III MINECO and Feder Funds (PI18/00858; PI18/00708; PI21/00953 and PI21/00315).

## Conflict of interest

The authors declare that the research was conducted in the absence of any commercial or financial relationships that could be construed as a potential conflict of interest.

## Publisher’s note

All claims expressed in this article are solely those of the authors and do not necessarily represent those of their affiliated organizations, or those of the publisher, the editors and the reviewers. Any product that may be evaluated in this article, or claim that may be made by its manufacturer, is not guaranteed or endorsed by the publisher.

## Glossary

**Table:**

^1^O_2_	singlet oxygen
ALA	aminolevulinic acid
BCC	Basal cell carcinoma
CAFs	cancer-associated fibroblasts
CCL5	Chemokine (C-C motif) ligand 5
CD	cluster of differentiation
CDK	cyclin-dependent kinase
CF	control fibroblastas
CTLA-4	cytotoxic T-lymphocyte-associated protein 4
CXCL12	C-X-C motif chemokine ligand 12
ECM	extracellular matrix
EMT	epithelial-mesenchymal transition
FAP	fibroblast activation protein
FGF	fibroblast growth factor
FOX	Forkhead box protein
GS	Gorlin Syndrome
HIF-1alpha	hypoxia factor 1 alpha
IFN-γ	Interferon gamma
IL	interleukin
MAL	methyl aminolevulinate
MAPK	mitogen-activated protein kinase
MC	mast cell
MCH-2	major histocompatibility complex 2
MDSCs	myeloid-derived suppressor cells
MMP	matrix metalloproteinases
mTOR	mammalian Target of Rapamycin
NF-κB	Nuclear factor kappa-light-chain-enhancer of activated B cells
NMSC	non-melanoma skin cancer
NO	nitric oxide
PDFG	Platelet derived growth factor
PD-L1	programmed death-ligand 1
PS	photosensitizer
ROS	reactive oxygen species
SCC	squamous cell carcinoma
scFv	sequence specific to FAP
SR-A	scavenger receptor A
STAT	signal transducer and activator of transcription
TAMs	tumor associated macrophages
TGFβ	transforming growth factor beta
TILs	tumor infiltrated lymphocytes
TLR	Toll like receptor
TME	tumor microenvironment
TNFα	Tumor necrosis factor
UVA	Ultraviolet A
VEGF	vascular endothelial growth factor
XF	xeroderma fibroblasts
XP	xeroderma pigmentosum
α-SMA	smooth muscle actin alpha.
